The article "Construction and Application of Talent Evaluation Model Based on Nonlinear Hierarchical Optimization Neural Network" was published in 2022. Journal: Comput Intell Neurosci.

# Construction and Application of Talent Evaluation Model Based on Nonlinear Hierarchical Optimization Neural Network

**DOI:** 10.1155/2022/6834253

**Published:** 2022-05-29

**Authors:** Xintian Pei

**Affiliations:** Jeonju University, Jeonju, Jeollabuk-do, Republic of Korea

## Abstract

Talent assessment attracts the attention of researchers because of its important influence on business management issues. The traditional talent evaluation model has high sample selection cost and large calculation volume ratio, so it has become an urgent problem to be solved. Based on the nonlinear hierarchical optimization neural network, this article improves the corresponding talent evaluation index system and builds a talent evaluation model on the basis of demonstrating the feasibility of using a nonlinear hierarchical optimization neural network for talent evaluation. This article conducts an empirical analysis on the talent evaluation model of the talent evaluation team members and designs a prototype system of the talent evaluation index system based on the nonlinear hierarchical optimization neural network. In the simulation process, MATLAB software is used to complete the program realization of the model, and the accuracy and feasibility of the model are verified by combining the case. Through the evaluation and research of the implementation personnel of the case enterprise, the enterprise talent evaluation based on the nonlinear hierarchical optimization neural network is demonstrated. The empirical results show that it is feasible and accurate to use the nonlinear hierarchical optimization neural network to evaluate the talent evaluation team. The comprehensive prediction accuracy rate of T-1 year is 88.5%, and the comprehensive prediction accuracy rate of T-2 year was 83.45%, which effectively promoted the evaluation of enterprise talents.

## 1. Introduction

With the increasingly intensified competition, marketing has become more and more important in business operations and has also received more and more attention from management. A successful marketing team plays a crucial role in talent assessment. However, talent evaluation relies on an excellent marketing team. Therefore, in order to gain a firm foothold in the fierce market competition and adapt to the environment of global economic integration and networking, an excellent marketing team must be formed [1]. How to make the marketing team members create maximum benefits in a fair and harmonious environment, it is very important to conduct a comprehensive, fair, and scientific talent evaluation for the marketing team members. The main purpose of talent evaluation of enterprise marketing team members is to establish an objective and fair talent evaluation system, on the basis of scientifically evaluating the contribution of talent evaluation team members to the enterprise, to establish an effective incentive mechanism, to cultivate talents, improve efficiency, and improve the overall competition of the company. It can promote the healthy growth of the enterprise and the marketing team, realize the standardized management of the team, and finally make the enterprise obtain greater profits [2–5].

Talent evaluation will be affected by many factors in the implementation process. The result is usually a multivariable, fuzzy, and complex nonlinear process, which is difficult to express through mathematical analytical expressions more accurately. Due to the inaccuracy of evaluation results, it greatly affects the role of talent evaluation in human resource management [6–9]. The nonlinear hierarchical optimization neural network technology is to imitate the neural structure and function of the human brain, which can deal with complex logical problems and realize nonlinear relationships. The biggest advantage of the neural network is that because of its strong versatility and very good self-learning and adaptability, it can simulate complex nonlinear relationships and be good at making decisions from uncertain or contradictory environments. Applying nonlinear hierarchical optimization neural network technology to talent evaluation to find out the nonlinear relationship between each index factor and evaluation results, avoiding manual determination of component proportions and calculation of correlation coefficients can make evaluation results more objective [10–13]. The construction of the model is to select a model suitable for the research object through research, and at the same time, it is necessary to verify the rationality of the constructed model through certain methods.

This article attempts to use the nonlinear hierarchical optimization neural network itself with the characteristics of parallel data processing, good fault tolerance, self-adaptation and self-learning, and good nonlinear functions, to systematically analyze the quality structure of enterprise personnel, and to construct a nonlinear hierarchical optimization neural network, to improve the evaluation method of enterprise personnel quality in order to reduce the deviation of evaluation results caused by subjective factors of evaluators. It is expected to obtain a general concise, objective and quantitative evaluation standards for the quality of enterprise personnel, and strive to improve the evaluation methods. The feasibility of applying the nonlinear hierarchical optimization neural network to the evaluation of personnel quality is demonstrated, and the principles and ideas of using the neural network to improve the evaluation method of enterprise personnel quality are introduced, and the evaluation model is established based on the nonlinear hierarchical optimization neural network model. The feature graphs generated by different convolutional layers in the full convolutional crowd counting network can be effectively fused so as to obtain richer hierarchical information and more detailed description features of the target scene. The neural network evaluation model is optimized for the nonlinear level, and the corresponding index system of enterprise personnel quality evaluation is established.

## 2. Related Work

The key talent index refers to the key index to measure the effect of enterprise strategy implementation. It is an operable index system generated by the decomposition of enterprise strategy layer by layer, and it is the basis of enterprise talent management. It sets, samples, calculates, and analyzes the key parameters of the information read into the information write end of some internal processes of the enterprise to obtain target-based quantitative management indicators. Its purpose is to establish a mechanism to transform corporate strategy into internal processes and motivations, continuously enhance the core competitiveness of the enterprise, enable the enterprise to achieve sustainable development, and avoid turning potential financial risks into actual economic losses; at the same time, it also helps managers to adjust business decisions in a timely manner, allocate enterprise resources more reasonably and effectively, and promote its long-term healthy development [14–17].

The management by objectives (MBO)-oriented talent management proposed by Lai et al. [18] mainly combines the evaluation process with the management process and has a good guiding role in the process of selecting key talent indicators that can achieve corporate goals and control the relevant key links of key talent indicators, so as to lead the enterprise forward under a correct and consistent guidance and, at the same time, stimulate the enthusiasm and creativity of employees, thus laying a solid foundation for the realization of the unity of operation and management within the enterprise. Guan et al. [19] believe that MBO-oriented talent management consists of four closely related parts, namely, planning, guidance, evaluation, and incentives. These four stages are combined with the four stages of management by objectives, execution, evaluation, and feedback, respectively. Therefore, the management by objectives method can enable employees to continuously work together to achieve corporate goals and achieve the improvement of personal ability and corporate efficiency.

Zhao [20] believes that the so-called quality evaluation is a set of standardized objective procedures used to determine the suitability of a particular person's job. It provides an accurate measure of a candidate's job-specific knowledge, skills, abilities, and attitudes against a set of predetermined criteria. According to the requirements, responsibilities, and needs of a specific job, the evaluation results of the participating evaluators are analyzed and evaluated. Chu et al. [21] believe that quality evaluation is to objectively formulate an individual's ability, work status, and adaptability, and to conduct an organized and realistic evaluation of an individual's personality, aptitude, habits, and attitudes, as well as the relative value of the organization, including evaluation sum of procedures, specifications, and methods. The large-scale parallel processing and storage, self-organization, self-adaptation, and self-learning capabilities of the nonlinear hierarchical optimization neural network make it suitable for, and especially suitable for, inaccurate and ambiguous information processing that needs to consider many factors and conditions at the same time. The nonlinear hierarchical optimization neural network has different advantages in different fields. In this article, the advantages of the neural network are applied to the evaluation of personnel quality to solve the difficult problems in the evaluation process and improve the objective and accurate evaluation results, performance, and evaluation speed, which are very feasible [22, 23].

## 3. Index Division of Nonlinear Hierarchical Optimization Neural Network

### 3.1. Nonlinear Hierarchical Optimization Neural Network Node Distribution

Calculating the comprehensive evaluation results of each nonlinear level optimization neural network object, once the comprehensive evaluation coefficient set *R* of membership degree is determined, the comprehensive evaluation result can be obtained by the following formula *W* = *R*, where “o” represents a certain fuzzy product operation selected according to the actual problem, also called operator. If only the key factors are considered, the operator of “or” type can be selected; the requirements of comprehensive consideration of various factors are used to judge things, it is necessary to use the “sum” type of operator: if both the overall consideration and the key points are to be taken into account, the *M* and *y* types of operators should be used at the same time. The comprehensive evaluation results under different operators are then synthesized at a higher level according to the multilevel model. At this time, the operator generally selects the operator corresponding to the comprehensive evaluation result with the largest weight [24, 25]:

(1) $$\begin{array}{c} \left\{\begin{array}{c} f\left(p,q\right)+f\left(p-1,q-1\right)<f\left(1,1\right),\\ f\left(s,t\right)+f\left(s-1,t-1\right)<f\left(0,0\right). \end{array}\right. \end{array}$$

In the comprehensive evaluation of the nonlinear hierarchical optimization neural network, it is a difficult part to determine the proportion of each factor in the U set, but it is also a very important part. The determination of the proportion of ingredients must be carefully and scientifically reliable. It should be as close as possible to the actual cause. Usually, the factor (indicator) that has a greater impact on the evaluation target has a larger weight; the factor that has a small impact on the evaluation target has a smaller weight:

(2) $$\begin{array}{c} this.\left(b\left(k,s\right)-b\left(k,t\right)\right)/\left(p\left(k,s\right)-p\left(k,t\right)\right),for\left(p<1\right). \end{array}$$

Each layer consists of several unit samples (nodes), and the information write value on each unit sample is determined by the information read value, activation information rate, and threshold. The learning process of the nonlinear hierarchical optimization neural network is as follows: after the learning information is provided to the nonlinear hierarchical optimization network, the information read-in information is propagated from the information read-in layer through the intermediate fuzzy layer to the information writing layer. The unit sample obtains the information reading response of the network, and then in the direction of reducing the error between the expected information writing and the actual information writing, the error information is reversely transmitted from the information writing layer through the intermediate fuzzy layer to the information reading layer, and layer by layer along the way and modify the connection information rate of each unit sample, so many cycles until the accuracy requirements are met, exit the loop, and store the connection information rate in each neuron of the network.

### 3.2. Change of Network Model Indicators

Each unit sample of the neural network can accept a large amount of information reading, and the relationship between information reading and information writing is nonlinear, so that unit samples can limit and influence each other. The constraint relationship between them ensures a nonlinear mapping of the entire network from information read to information write. From a global perspective, the simple addition of the local performance of the network is not equivalent to the overall performance. The unit samples and their connections in Figure 1 only represent a part, not a complete specific concept. The distributed comprehensive effect of each unit sample is expressed.

According to the previous discussion, in order to let business leaders know clearly what aspects to measure and evaluate candidates during the assessment, so as to make an objective and accurate prediction on the talents of candidates in their applied positions, a talent evaluation index system based on the nonlinear hierarchical optimization neural network is established, and the measurement methods of each nonlinear hierarchical optimization neural network index are given, and in-depth exploration and definition are carried out from the perspective of quantitative analysis:

(3) $$\begin{array}{c} \langle \begin{array}{c} k\text{network }\left(p,c_{a-b}^{a+b}\right)=f\left(n,w^{\prime }\left(m,n\right)\right),\\ k\text{network }\left(c,p_{a-b}^{a+b}\right)=f\left(m,w\left(m,n\right)\right). \end{array} \end{array}$$

This article uses the neural network toolbox in MATLAB to learn, train, and simulate the nonlinear hierarchical optimization neural network, and the main points of the program debugging method. Now, the ten candidates for the position of implementation personnel are evaluated, and the score values of 16 secondary indicators are given. The specific algorithm has been introduced above and will not be repeated here. Through the evaluation model we constructed, the comprehensive score value *v*′ of the ten candidates is obtained. At the same time, we also give the comprehensive score value *v* obtained by the fuzzy comprehensive evaluation method. By comparison, we can see that the trained nonlinear hierarchical optimization neural network reaches the expected error level.

### 3.3. Nonlinear Hierarchical Optimization Neural Network Component Proportion Recursion

During network training, in order to ensure that the data are of the same order of magnitude, it is necessary to perform certain preprocessing on the input of the neural network and the information written into the data, which can speed up the training of the network. There are three preprocessing methods provided in MATLAB: normalization processing (change each group of data into a number between (−1, 1). The information rates involved are PREMNMX, POSTMNMX, TRAMNMX), normalization processing (change each group of data into data with a mean of 0 and a variance of 1. The information rates involved are PRESTD, POSTSTD, TRASTD), and principal component analysis (perform orthogonal processing to reduce the dimension of the information read into the data. The information rates are PREPCA, TRAPCA). In the empirical research, this article normalizes the information read-in data involved and performs the data information read-in operation in Figure 2.

The working group is mainly composed of personnel from the Human Resources Department who have been trained in the construction of the nonlinear hierarchical optimization neural network. At the same time, direct supervisors, senior technical personnel, and senior management personnel of each department are required to participate in order to cooperate with the construction of nonlinear hierarchical optimization neural network construction. As long as they have received the necessary training, they can quickly and accurately establish their competency characteristics model. It is very practical and has application value, so their participation is very necessary.

### 3.4. Evaluation Basis of Network Data

The neural network can realize the storage and memory of information by using its own network structure. These memories are stored in the connection information rate of the unit sample in a distributed storage manner, so the information content cannot be found only from a single information rate. This is also the reason why neural networks have good fault tolerance. The good fault tolerance of neural network enables it to perform information processing such as feature extraction, memory restoration, and cluster analysis and is also good at pattern recognition such as pattern association and pattern classification. When the hardware or software of the network is abnormal in a unit sample, the good fault tolerance also enables the entire network to still work normally. On the other hand, when the information read into the information is inaccurate or relatively vague, the associative memory function of the neural network in Figure 3 enables the neural network to still associate the complete image stored in the memory.

In the training process of designing the network, the optimal expected error should be sought through comparative training. The so-called “optimal” is determined relative to the number of nodes in the fuzzy layer, because the smaller expected error value is obtained by increasing the number of nodes in the fuzzy layer and the training time. On the basis of sufficient investigation and interviews, this project has repeatedly demonstrated and determined its evaluation indicators, and formulated appropriate evaluation scales and methods for each evaluation indicator. Finally, the evaluation indicators of the *T* Group's personnel quality evaluation project were generally determined into five major items, each of which was divided into various quality contents to be tested separately. The most realistic evaluation results can be obtained.

## 4. Construction of Talent Evaluation Model Based on Nonlinear Hierarchical Optimization Neural Network

### 4.1. Nonlinear Hierarchical Optimization Neural Network Data Feature Extraction

The newff data eigenvalue is used to create the information rate of the nonlinear hierarchical optimization neural network. The information rate can also determine the number of layers of the network and the number of neurons in the fuzzy layer. The information rate has six information read-in parameters: the range of the information read-in vector, the network structure, the transform information rate of each layer, the training algorithm information rate, the learning information rate, and the performance information rate. The information write parameters are built-in nonlinear hierarchical optimization neural networks. First, we make the number of fuzzy layer units variable or put enough fuzzy layer unit samples, and eliminate those ineffective unit samples through learning until they cannot be contracted. Similarly, a relatively small number of unit samples can also be put in at the beginning, and after a certain number of learning, if unsuccessful, the number of unit samples can be increased until a reasonable number of fuzzy layers is reached.

Using the yam information rate, the network can be trained with information data after initialization. The training network in Figure 4 has a gradual mode and a batch mode. The progressive mode is to read information one learning information at a time. Each time the information is read, the information rate and threshold will be changed according to the performance information rate, while the batch mode is to adjust the information rate and threshold after all the information is learned. In the batch mode, there is no need to set the training information rate for the information rate and threshold of each layer, and only one training information rate needs to be set, which is more convenient than the gradual change mode.

In this case, the knowledge and skills factor information in Table 1 is read into 4 nodes; the behavior ability factor information is read into 6 nodes; the personal style factor information is read into 4 nodes; the motivation factor information is read into 4 nodes. The number of read-in layer nodes is 2; after repeated experiments in this article, the number of unit samples of a single fuzzy layer is finally determined to be 4, and according to the previous design of the nonlinear hierarchical optimization neural network, the information write-in layer unit sample is set to 1 individual:

(4) $$\begin{array}{c} u\left(a,b,c\right)=\left[\begin{array}{ccc} t\left(a\right) & t\left(b\right) & t\left(c\right)\\ t\left(a-1\right) & t\left(b-1\right) & t\left(c-1\right)\\ t\left(a-t\right) & t\left(b-n\right) & t\left(c-t\right) \end{array}\right]. \end{array}$$

The learning rate of the data eigenvalues determines the amount of information rate change produced in each loop training. If the learning rate is too large, the system will be unstable; if it is too small, the training time will be too long and the convergence speed will be slowed down, but it is easy to find the minimum error value. On the other hand, many improved training algorithms can only use batch mode. Among them, Si represents the number of unit samples of the *i*-th layer network, the network has a total of N layers, *i* is the transformation information rate of the *i*-th layer network unit sample, BTF is the information rate of nonlinear hierarchical optimization training algorithm, BLF is the learning information rate, and PF is the performance information rate.

### 4.2. Topology of Talent Evaluation Model Index System

In the process of talent evaluation using the nonlinear hierarchical optimization neural network method, it is also necessary to artificially determine various evaluation factors in the indicators. Therefore, in the process of talent evaluation, the richer the evaluator's qualifications and experience, the stronger the ability to extract data and information, and themore objective the evaluation result is. This kind of thinking method of the evaluator's brain is the operation principle of neural network technology; that is, try to carry out evaluation through effective experience and relevant standards set by the enterprise, make the evaluation process programmatic and scientific, and minimize the subjective arbitrariness:

(5) $$\begin{array}{c} \underset{x⟶\infty }{\lim}\frac{z\left(x,t\right)+z9x,t-x}{z\left(t^{\prime },t\right)}\underset{x⟶\infty }{\lim}\left(x,t\right)>0. \end{array}$$

The nonlinear hierarchical optimization neural network is just a method that can deal with complex nonlinear problems in complex environments such as ambiguous, uncertain, and incomplete information. The self-learning ability of the network makes the traditional expert system technology application, the most difficult way of knowledge acquisition, to be transformed into the structure adjustment process of the network, so it can make reasonable judgments on complex problems.

After the information is collected, the information in Figure 5 should be sorted out, and a transitional nonlinear hierarchical optimization neural network should be established. In the stage of establishing the transitional competency model, the information collected earlier should be classified according to different job categories, and then, the neural network classification should be optimized according to the four types of nonlinear levels set in this article and then analyzed and recorded. Next, compare the occurrence frequency and related degree statistical indicators of the element indicators of the excellent group and the ordinary group, find out the common and different characteristics of the two groups, and estimate the approximate proportion of each feature group according to the degree of frequency concentration. It is also possible to first classify the neural network according to the four types of nonlinear hierarchical optimization and then classify it according to the position:

(6) $$\begin{array}{c} w\left(m,n\right)=\left\{\begin{array}{c} x\left(n+1\right)+\frac{x\left(n\right)}{\left(n+1\right)},n\leq m,\\ x\left(n+1\right)-\frac{x\left(n\right)}{\left(n-1\right)},n>m \end{array}.\right. \end{array}$$

The learning rate, that is, the step size, is a constant in the standard nonlinear hierarchical optimization neural network. For the standard nonlinear hierarchical optimization neural network algorithm, it corresponds to a suitable learning rate, which is usually a constant. But it is very difficult to determine a fixed learning rate in the actual calculation process. If the learning rate is too small, the training time will increase, which will affect the convergence, and the minimum error value cannot be guaranteed, but if the rate is too large, the neural network may collapse. Usually, the selection range of the learning rate is 0.01–0.8. In this article, the learning rate is set as 0.0l when constructing the nonlinear hierarchical optimization neural network of talent evaluation team.

### 4.3. Network Model Information Rate Transfer

The nonlinear hierarchical optimization neural network is trained by a mentor. By adjusting the connection information rate and threshold of each layer, the network learns the rules expressed by the training information. Using the neural network toolbox under MATLAB to train the network needs to provide training information to the network. The training information is composed of the information read-in information write-in pair (*x*, P), where *x* is the information information read-in vector, and *y* is the information information write-in vector. In the application of the neural network toolbox, *P* is often used to represent the input information vector and *f* to represent the information written into the information vector. In this article, *p* represents the index value of each nonlinear level optimization neural network, and *t* is the comprehensive score:

(7) $$\begin{array}{c} y\left(w\left(r\right),r\right)=\langle \begin{array}{c} |\sum_{r-1}\frac{n}{\left(w-r\right)!-r!},r>n\\ |\frac{w!}{r!\left(n-r\right)!}-r,r<n \end{array}.. \end{array}$$

This program is oriented to the three-layer nonlinear hierarchical optimization network learning algorithm, and the user can freely customize the structural parameters and learning parameters of the neural network shown in Figure 6: structural parameters such as the number of information read-in units, the number of information write units, the number of fuzzy layer units, training algorithms, and activation information rates; and learning parameters such as system accuracy, maximum training times, and step size. If the user does not set the learning parameter, the default value will be used.

In the design process of the nonlinear hierarchical optimization neural network, it needs to have good generalization ability; that is, the designed system needs to have strong adaptability to fresh information. In general, the generalization ability is determined by three factors, such as the complexity of the problem, the complexity of designing the network model, and the amount of learning information. Therefore, in the process of constructing the talent evaluation model of the talent evaluation team based on the nonlinear hierarchical optimization network neural network, it is necessary to consider the number of layers, the selection of the proportion of components, the learning rate, the number of unit samples, errors, and other related factors.

In the process of neural network training, the transmission activation information rate is the key link of training, and the characteristic of transmission information rate requires that the information read data of its information are in the [0, 1] interval, so the network training required in Table 2 must be it. The original information data are preprocessed and converted into data distributed in the range of [0, l], which is the basic work of the network model training process. The specific method of preprocessing depends on the order of magnitude of the original data, which is determined according to the maximum value of each information read in the data.

## 5. Application and Analysis of Talent Evaluation Model Based on Nonlinear Hierarchical Optimization Neural Network

### 5.1. Data Collection and Analysis of Nonlinear Hierarchical Optimization Neural Network

In general, the number of unit samples of the fuzzy layer is determined by the network convergence performance and the fluctuation of the information rate. That is, the loss is calculated separately in each stage of the network, so as to ensure the normal parameter update in network training and solve the problem that the over-deep network is difficult to optimize. Too much or too little number of unit samples is not suitable for the model, and more fuzzy layer nodes can bring better performance, but it may lead to too long training time, and it is difficult to use an ideal expression to represent the number of fuzzy layer unit samples, but a suitable number of fuzzy layer unit samples can be selected by combining experience and repeated experiments:

(8) $$\begin{array}{c} \frac{\text{d}p\left(x\left(i\right),y\left(i\right)\right)}{\text{d}p\left(x\left(i\right)\right)-\text{d}p\left(y\left(i\right)\right)}-\frac{k\left(x,a\right)}{k\left(x,b\right)}=0. \end{array}$$

Therefore, in the selection process of the initial value, it should be noted that the proportion of the initial component is generally a random number as small as possible, so that the state value of each unit sample can be as close to zero as possible when it is accumulated, ensuring that the unit the samples all fall in the position where the derivative of the transmission information rate is the largest; that is to say, the adjustment of the proportion of the connection component of the unit sample is carried out at the place where the sigmoid activation information rate changes the most. Typically, the initial information rate of Figure 7 is typically a random number between 0 and 1.

The horizontal extension of this model is the analysis of the motion matrix of complex systems. The vertical extension is combined with the CRP paradigm, Proposition 3, Proposition 4, Proposition 5, and Proposition 6 to propose a three-dimensional coefficient set model. Since the CRP model serves the strategic management of airport enterprises, the implementation effect of the strategy formulated by using this model will be the only criterion for testing the model and also the main basis for strategic adjustment according to environmental changes.

### 5.2. Simulation Realization of Talent Evaluation Model

In order to make the operation interface of the talent evaluation model friendly and operable and use high-quality computer programs to assist the application research of theoretical exploration, this article has carried out a lot of work in the realization of neural network software, and designed and developed a neural network based on Visual C++ simulation program. The number of unit samples of the information read-in layer depends on the dimension of the information read-in vector. According to the previously defined marketing team member talent evaluation index system, there are a total of 21 indicators including psychological quality, sense of responsibility, and spirit of cooperation.

Therefore, the number *n* of neurons in the information read-in layer is determined to be 21. The number of unit samples in the information writing layer is determined by the information writing results of the actual problem. In the evaluation model of this article, it is hoped that a comprehensive talent evaluation result can be obtained through each individual indicator, and the comprehensive talent evaluation result of the marketing team members is used as the result. Since the information is written into the signal, the number *m* of unit samples of the information written layer is 1.

For a large enterprise, there are many positions involved, so the records are generally classified in the form of codes. In the process of coding, the coding should not only reflect the category of the nonlinear hierarchical optimization neural network itself, but also reflect the targeted position category, so that it is easy to find and use in the process of later induction and correction. Finally, all codes are sorted out, the same or basically similar nonlinear hierarchical optimization neural networks are merged, defined, and coded again, and a general description of each nonlinear hierarchical optimization neural network is shown in Figure 8. The degree has a detailed description of the level.

Through data analysis, it can be judged which nonlinear hierarchical optimization neural network in the preliminary nonlinear hierarchical optimization neural network is more important. In the analysis, the average and frequency are generally used to measure respectively. First of all, the evaluation level of the nonlinear hierarchical optimization neural network is divided into very necessary, necessary, useful but unnecessary, and unnecessary, and attached with 4, 3, 2, and 1 points, respectively, and the average value is each nonlinear hierarchical optimization neural network for the average score of the network at the time of rating. Frequency is the number of times these four rating levels occur in a nonlinear hierarchical optimization neural network.

The final conclusions are determined by analysis of statistical techniques (*t*-test, standard deviation analysis, variance analysis). Through data analysis, nonlinear hierarchical optimization neural network items that are not related to effectiveness can be removed; inaccurate feature items can be corrected; missing feature items can be added; and finally, the model construction can be completed.

### 5.3. Example Application and Analysis

The nonlinear hierarchical optimization neural network index of the talent evaluation model mainly includes the first two levels of the nonlinear hierarchical optimization neural network, namely, knowledge and skills. The score level of the candidate can be more accurately determined according to the mastery of the actual knowledge and skills of the candidate; that is, the absolute quantification of the nonlinear hierarchical optimization neural network can be directly carried out, such as the professional knowledge level, skill level, foreign language, and computer level of the position to be applied for by the candidate:

(9) $$\begin{array}{c} \sum_{i,s<t-i}\frac{w\left(i,j\right)}{w\left(i,j\right)-1}=\left[\begin{array}{cc} w\left(i,j\right) & 1\\ 1 & -w\left(i,j-1\right) \end{array}\right]. \end{array}$$

Different enterprises and different positions need to establish different nonlinear levels to optimize the neural network assessment indicators according to their own conditions. At the same time, it is also necessary to set the corresponding evaluation level, and the setting method of the level can refer to the subjective nonlinear hierarchical optimization neural network.

When designing the BARS scale, it is now common practice to develop a 50-level scoring table for each nonlinear hierarchical optimization neural network. Within each level, accurately list the behavioral indicators on that level. Accuracy here means that the description of the behavior should be accurate and specific on the one hand; on the other hand, the given behavior index should meet the requirements of the degree of nonlinear hierarchical optimization neural network at this level. For the level defined by each behavior, four elements can be considered, namely, serial number, score, qualitative description, and specific behavior indicators. For example, when performing the measurement of Figure 9 on the nonlinear hierarchical optimization neural network of “activeness,” it can be set to five levels, and the second and fifth levels can be programmed in this way.

It can be seen that the correlation between the indicators is relatively large, which is suitable for principal component analysis. The KMO test result of the information is 0.643, indicating that the correlation between variables is relatively large, and the Sig value is less than 0.05, indicating that there is a correlation between the 28 variables, and the principal component analysis method can be used to analyze the selected variables. For a particular position, candidates are required to have several nonlinear hierarchical optimization neural network metrics in different categories. Each nonlinear level optimization neural network index has a different degree of influence on high-caliber talents, so it is necessary to set the proportion of components for different nonlinear level optimization neural network to measure its importance and influence. At the same time, the factor common degree results reflect the common degree of 8 principal components of 28 variables. It can be seen that most of the common principal components of the 28 early warning indicators are above 0.8, indicating that the 28 primary early warning indicators are well explained by the 8 principal components.

## 6. Conclusion

This article first integrates AHP and fuzzy comprehensive evaluation technology to provide relatively effective training information for nonlinear hierarchical optimization neural network and then builds a nonlinear hierarchical optimization neural network evaluation model for enterprise talent evaluation. The trained nonlinear hierarchical optimization neural network is used to comprehensively evaluate the candidates, and the size of the comprehensive evaluation value can objectively and accurately predict the candidate's future work talent level. At the same time, on the basis of analyzing the shortcomings of traditional talent evaluation, it is pointed out that the talent evaluation based on the nonlinear hierarchical optimization neural network can enable enterprises to obtain talents for business talents, and then, the talent evaluation index system based on nonlinear hierarchical optimization neural network is constructed. Accurately, they reflect the nonlinear hierarchical optimization neural network that highly talented employees should have; in the quantification method of nonlinear hierarchical optimization neural network indicators, different measurement methods are given from the subjective and objective perspectives, thus ensuring the accuracy of quantitative analysis; combined with the construction of the nonlinear hierarchical optimization neural network index system of the individual enterprise implementers, the general methods and steps of establishing the nonlinear hierarchical optimization neural network index system are given. Aiming at the fuzziness of nonlinear hierarchical optimization neural network indicators and the subjectivity of current evaluation methods, a comprehensive evaluation model integrating neural network technology is proposed. In addition, as the network deepens, it is easy to disappear the gradient in the process of back propagation, so we adopt an objective function to optimize the relay supervision at each stage. The evaluation model can not only weaken the human factors in the determination of the proportion of components, but also has the functions of intelligence, self-adaptation, and self-learning and can be continuously optimized by accumulating evaluation experience.

## Figures and Tables

**Figure 1:** The distribution of network model index changes.

**Figure 2:** Node distribution of the nonlinear hierarchical optimization neural network.

**Figure 3:** Histogram of network data evaluation.

**Figure 4:** Nonlinear hierarchical optimization neural network data fitting distribution.

**Figure 5:** Two-dimensional distribution of the indicator system of the talent evaluation model.

**Figure 6:** Information rate transfer polarization distribution of the network model.

**Figure 7:** Statistical distribution of the nonlinear hierarchical optimization neural network data.

**Figure 8:** Structure distribution of the talent assessment model.

**Figure 9:** 3D analysis of principal components of nonlinear hierarchical optimization neural network indicators.

**Table 1:** Information data training after initialization.

Information data threshold	Training mode behavior ability factor
S (sno, sname, password)	Using the yam *x*(*n*+1) − *x*(*n*)
C (cno, cname, ctine, cplace, tno)	lim_*x*⟶*∞*_*z*(0, *t*) information rate
T (Tno, Tname, password)	The number of *b*^2^ − 4*ac*
Sno char (10) foreign key references S(Sno),	The network can *w*(*r*)
Cno char (10) foreign key references S(Sno),	The knowledge and (*w* − *r*)!−*r*!
Tname char (10),	*t*(*b* − *n*) be trained
Password char (10)	Unit *u*(*a*, *b*, *c*) samples
Public void keypressed (e) {	With *n*, *r* ∈ *C*(1,1) information data
Plane.key-released-control-direction (e);	*knetwork*(*p*, *c*_*a*−*b*_^*a*+*b*^) after initialization

**Table 2:** Nonlinear hierarchical optimization network sample sequence.

Network sample	Evaluation a	Evaluation b	Evaluation c	Evaluation d
Np 1	1.3	1.36	1.42	1.48
Np 2	0.73	0.75	0.77	0.79
Np 3	0.16	0.14	0.12	0.1
Np 4	0.41	0.47	0.53	0.59
Np 5	0.98	1.08	1.18	1.28
Np 6	1.55	1.69	1.83	1.97
Np 7	2.12	2.3	2.48	2.66

## Data Availability

The data used to support the findings of this study are available from the corresponding author upon request.
